The article "Extraction and Analysis of Foot Bone Shape Features Based on Deep Learning" was published in 2022. Journal: Comput Math Methods Med.

# Extraction and Analysis of Foot Bone Shape Features Based on Deep Learning

**DOI:** 10.1155/2022/2372160

**Published:** 2022-08-10

**Authors:** Yue Ma, Zhuangzhi Zhi

**Affiliations:** ^1^School of Forensic Science, Criminal Investigation Police University of China, Shenyang 110854, China; ^2^Key Laboratory of Impression Evidence Examination and Identification Technology, Ministry of Public Security, Shenyang 110854, China; ^3^School of Medical Instrument, Shenyang Pharmaceutical University, Shenyang 110016, China

## Abstract

With the rapid development of artificial intelligence, more and more researchers and research institutions begin to pay attention to the bone feature recognition field. Human bone movement is very complex, and human bone shape recognition technology can be widely used in medical treatment, sports, and other fields. At present, there are mainly two kinds of methods for extracting the shape features of human foot bone based on optical image acquisition technology and sensor information perception technology. However, due to the interference factors such as target posture change, camera shake, and individual behavior differences, it is still a very challenging task to design a robust algorithm for extraction and analysis of foot bone shape features. In recent years, convolutional neural network- (CNN-) based foot contour feature recognition methods emerge one after another and have made breakthrough progress. How to use and how to fully explore the potential relationship of various characteristics contained in the foot bone data and how to enhance the robustness of view changes and other aspects need to be further studied. In this context, this paper proposed an improved CNN model, which not only has the capability of deep feature extraction of the CNN model but also can obtain the optimal model parameters with the combination of particle swarm optimization algorithm. The effectiveness of the proposed method in the extraction and analysis of foot bone shape features is verified in the simulation experiment.

## 1. Introduction

With the development of science and technology, human body skeleton recognition in the field of artificial intelligence has been a very hot research topic, and the position of the human skeleton is extracted and identified in the image, so as to track the human body and identify, analyze, and judge the human actions. Human motion recognition is a subject involving many fields [1, 2]. Nowadays, people can sense and capture movement information through the eyes, head, ears, and other organs, extract the obtained information in the brain, and finally input it into the computer for movement recognition and judgment. The human action recognition algorithm imitates the human action recognition process, automatically detects the human action from the action sequence data collected by various sensors, analyzes the human action, and deduces its semantic information. However, the law of human movement is highly complex, especially the simulation of human movement coordination mechanism being very difficult, so the development of science and technology is still unable to generate very realistic movement data based on algorithms or other ways [3]. Motion capture technology still plays a very important role in medical film and television scenes and can overcome the problems of high complexity and high nonlinear simulation mechanisms.

The article "Extraction and Analysis of Foot Bone Shape Features Based on Deep Learning" was published in 2022. Journal: Comput Math Methods Med.

Motion recognition technology based on human bone points can be widely used in public security, intelligent home, wisdom classroom, and other fields. (1) Public security: this includes airports, stations, and other crowded public areas, for the installation of monitoring equipment systems [4, 5]. Once suspected criminals are found and some unconventional behaviors are identified by the system, the public security organs can get alarm information and immediately send police to control criminals, avoid the spread of criminal activities, and protect people's personal and property safety. Human motion monitoring technology based on bone recognition can expand the early warning range of public monitoring and relieve the pressure of public security. (2) Smart home: human motion recognition systems can also be combined with the Internet of Things devices, becoming a basic technology in smart homes. Intelligent control of household equipment can be realized by recognizing human movement. It also can realize home monitoring; once the elderly and children fall, it will immediately send a message to inform the family to deal with it. Once there is an intruder, it can also carry out intelligent alarm tracking, to ensure the safety of the family property. (3) Intelligent class: students' performance and behaviors in class can be classified and counted to analyze the teaching state and classroom atmosphere in each period of class. Schools and teachers take it as a reflection of teaching quality and then carry out teaching policy improvement to improve teaching quality.

Among them, the traditional target detection algorithm, the recognition, detection, and tracking of human bone movement belongs to the low-level processing mode of machine vision, and this kind of algorithm does not need to carry out a large number of training data sets. The recognition of human bone movement is a more advanced stage. The detection of the action of the testee is the key to visual processing. Many scholars have proposed mature algorithms for the solution of action recognition and detection. In the traditional field, human target detection methods include background subtraction, frame difference, and optical flow. These methods are mainly used for tracking through matching and motion characteristics. Using deep learning, the method of human-computer interaction is in the advanced processing stage. The human motion detection and motion analysis-related technologies of this kind of algorithm are in the hot spot of exploration and research [6]. In the traditional field, human target detection methods include background subtraction, frame difference, and optical flow. These methods are mainly used for tracking through matching and motion characteristics. In using deep learning, the method of human-computer interaction is in the advanced processing stage. The core technology hidden behind this kind of human motion detection and analysis method is the hot spot and difficult point of academic and industrial research. Researchers collect bone characteristics from smart devices to monitor human health and physical training and track the lives of older adults. Intelligent devices to detect bone features have been widely used in people's daily life and social production. Using deep learning, the human-computer interaction method for bone feature detection and analysis of the relevant technology is the focus of exploration and research [7].

The article "Extraction and Analysis of Foot Bone Shape Features Based on Deep Learning" was published in 2022. Journal: Comput Math Methods Med.

In human life activities, walking is the most common behavior of the human body, and the body posture change presented in the process of walking is called gait. It is deceptively simple but involves the precise coordination of multiple tissues and organs throughout the body [8]. Among them, the brain generates the intention to walk, and the central nervous system decomposes the intention and transmits control information to the muscle tissues involved in the movement. Each muscle tissue generates joint torques through contraction, thus driving the limb bones to complete the walking action. Obviously, in this series of information transmission and drive control process, gait contains abundant mechanism characteristics and life system mystery of the human body. The in-depth analytical study of human foot bone movement and the discovery of useful characteristic information have important guiding significance for the development of lower limb exoskeleton robot project and the application based on foot bone characteristics. For a long time, people are constantly exploring and studying their own foot bone movement [9]. Humans have been studying their own walking movements for centuries, but due to the limitations of science at the time, the earliest studies of foot bone characteristics were only a few lines of written records. Subsequently, with the advent of sensors, computers, and other modern instruments, the research on foot bone characteristics has gradually become scientific. At the same time, the in-depth study of foot bone also promotes the rapid development of information science, which is closely related to human biology. Based on the previous theoretical research and coupled with advanced instruments and equipment, now, the study of foot bone characteristics can be more and more in-depth [10].

The article "Extraction and Analysis of Foot Bone Shape Features Based on Deep Learning" was published in 2022. Journal: Comput Math Methods Med.

As a key technology in artificial intelligence, feature fusion technology has great innovation space and application value, attracting more and more enterprises and research institutions. From the perspective of motion recognition, human skeleton recognition can be roughly divided into posture data acquisition, skeleton dynamic data acquisition, and key posture mining. To meet the requirements of personal information security, the foot bone movement in posture characteristics is regarded as a collection of hard connected segments between the nodes of the human physiological skeleton. At present, various organizations and well-known universities have spent a lot of energy and time on the research of this technology [11, 12]. In order to give full play to the advantages of depth image and bone data, the depth feature is combined with the foot bone feature for human behavior recognition. The method of human behavior extraction based on feature fusion is studied to capture behavioral cues in depth images and extract the combined features of human behavior. Then, using skeletal data to extract various features of foot bone shape achieves results only related to behavioral distribution, but it takes a long time. Some scholars also proposed the iterative learning control algorithm to track human foot bone joint and knee feature extraction method, combined with human lower limb structure analysis, to establish the dynamic model of lower limb exoskeleton robot [13]. Therefore, how to use the deep learning model to extract and analyze the shape features of human foot bone has important theoretical value and practical application prospect. Here, the layout of this paper is the following: Section 2 gives the related works; then, the proposed method is shown in Section 3. After that, the simulation results are introduced in Section 4. Finally, Section 5 concludes the article.

## 2. Related Work

Under the guidance of image processing and machine vision technology, the development of foot bone feature recognition technology not only has universal market value and huge economic value in medical monitoring, elderly monitoring, and motion analysis but also has academic research significance [14, 15]. Due to the high research value of human skeleton recognition in many aspects, a large amount of investment has been stimulated at home and abroad. In recent years, whether the government or enterprises, people from all walks of life in the field of human behavior identification investment in a large number of human, financial, and material resources so far have made rich achievements. Human motion recognition can extract the key features of human motion by obtaining the video sequence of human motion. After years of research, researchers have conducted an in-depth exploration of human motion recognition algorithms, formed a number of research directions, and achieved a lot of valuable results. According to the different human motion features adopted by the algorithm, human motion recognition can be divided into the following categories. The following is a brief introduction based on the existing research results.

(1) Foot bone feature recognition is based on human body structure features. The human body structure can be expressed as the trunk and limbs connected by joints. An action video sequence can be seen as the combination of different human poses generated by the relative displacement of different body parts in a certain time range. The motion representation features are extracted from the three-dimensional bone point information of the human body. The common steps include human motion detection, bone point information extraction, bone point information description, extraction of relevant features, and classification of human motion. (2) Foot motion recognition is based on global features. Global feature refers to the feature that represents the action in the whole sequence, which is usually the spatial change of the whole sequence with spatiotemporal information. The first is to identify the region of interest, the use of target detection, and other ways to identify the human body region, and then, through the region of the posture trajectory and other related information, the human movement of the region of interest is described and finally realizes the human bone movement recognition. (3) Human foot bone motion recognition is based on local structural features. Local features of the human body refer to the local parts of the body that change significantly, such as the arm and neck, through the characteristics of these parts to characterize the whole movement. The motion recognition algorithm based on local structural features firstly extracts the human motion features from video sequences, then describes the feature points with appropriate descriptors, calculates the local body features, and finally establishes a classifier to recognize human actions [16, 17].

The article "Extraction and Analysis of Foot Bone Shape Features Based on Deep Learning" was published in 2022. Journal: Comput Math Methods Med.

Motion captures data in animation; film production has the real nature of the task action, can make the movie role more vivid, and is the basis of high-quality animation and special effects. And the motion data in this application field will still be an important part, but motion capture equipment is expensive, the motion capture process is complex and tedious, and there is motion data processing workload and other shortcomings. In order to improve the utilization of motion capture data, in recent years, human motion data prediction, motion sequence fragment transition, and other technologies emerged. The main prediction methods of human movement data include deep learning models based on adversarial neural network and recurrent neural network as well as traditional methods [18]. The transition technology models of motion sequence fragments mainly include probability statistics, motion graph, and deep learning. For the transition model of motion sequence fragments, in order to make full use of the reusability of motion data, several short or moving sequence fragments can be spliced together to generate a long moving sequence with complex semantics. If the sequence of walking and running, which have different postures and semantics, is directly spliced together, there will be a very stiff sliding step and space jump of movement track, and the human eye is very sensitive to this difference. Compared with foreign countries, domestic research on human behavior recognition started a little later, but many domestic universities and research institutions have made some achievements in this area [19]. At present, domestic research institutions have gradually reached the development level of the foreign research field, and some of them can be used as commercial systems. Some famous conferences and international authoritative journals have opened relevant columns on human bone behavior recognition, which provides a platform for communication for the majority of enthusiasts and will greatly promote the rapid development of behavior recognition. Major conferences and journals include PAMI (IEEE Transactions on Pattern Analysis and Machine Intelligence), Image and Vision Computing (IVC), and Computer Vision and Image Understanding (CVIU). Although the above methods have achieved a lot in the extraction and analysis of foot bone shape features, these methods are all shallow models, and the relevant research on the deep learning model will be introduced next.

The deep learning method is the preferred model for image processing, image recognition, and classification system [19]. Neural networks are widely used in recognition systems, natural language processing, and recognition. Compared with traditional detection methods, the main advantage of the neural network is that it can be detected automatically without any human supervision and it also has high computational efficiency. Its algorithm using the convolution layer and pooling layer is very simple and can be applied to other instances only by adjusting its parameters appropriately. This enables the neural network model to run on other devices, which makes the neural network have universal applicability. However, the convolutional neural network (CNN) algorithm cannot deal with continuous time series, which greatly increases the limitations of the convolutional neural network algorithm. Among deep learning algorithms, the most mature algorithm at present is the CNN algorithm, which is widely used and can be said to be the most popular deep learning architecture at present, which greatly improves the huge popularity and effectiveness of deep learning [20]. At present, human skeleton motion detection is most widely used by machine vision technology and digital image processing technology. Deep learning can directly learn two-dimensional images without changing the structure of image nodes, which can greatly reduce a lot of manual processing of image input and can achieve comprehensive automation without excessive human participation, and the learning process is completely completed by the system itself. Deep learning has been widely used in various fields of image recognition, such as target line recognition of license plate recognition of face recognition of wood and so on. The deep learning method not only has good learning ability but also can accurately extract the recessive features that reflect the essence of input sequence and accurately identify detection objects [21]. Therefore, it has the characteristics of fast discrimination, high cost performance, simple operation, and safety, which greatly improves the process of automatic recognition of human movements. Therefore, it can be applied to the research of foot bone feature extraction and recognition.

The article "Extraction and Analysis of Foot Bone Shape Features Based on Deep Learning" was published in 2022. Journal: Comput Math Methods Med.

At present, the traditional bone feature recognition methods include the optical flow method and frame difference method, but these methods cannot complete the detection and recognition of complex actions, and their low efficiency and high misjudgment rate cannot meet the needs of the market. In order to enable intelligent equipment to efficiently identify human movements and check the standardization of movements, deep learning can be used for processing [22]. The combination of human behavior recognition and human movement detection methods will greatly improve the accurate recognition of human bone movement, promote the development of factory movement detection related fields, and ultimately improve the economic benefits of enterprises. Human bone feature recognition and analysis of human activities have always been the field of computer vision, machine learning, and artificial intelligence. Human motion analysis is a complex video-based processing process that captures both single frame position information and dynamic motion features. It can realize automatic understanding and analysis of data by computer through human-computer interaction and establish relationships between data related to low-level and high-level semantic operations. However, in real-world application scenarios, surveillance cameras usually have multiple perspectives, which will result in great differences for intelligent devices such as computers to understand and process scene content from different perspectives. At the same time, it is urgent to evaluate the mobile status of equipment with secure and real-time performance [23]. Therefore, the robustness, accuracy, and effectiveness of the method to evaluate human skeletal state are important challenges for future research. In order to realize the spatial information analysis of the skeleton by computer, some scholars proposed the ST-GCN network. ST-GCN represents the skeleton array of the spatiotemporal graph network (ST-GCN) on the spatiotemporal graph network (ST-GCN) and designs the motion recognition model by extending the graph network. The model is based on the skeleton diagram, and each node is associated with the joints of the human body. This model is mainly divided into two types, and each model has an edge structure. An edge corresponds to the natural connection of every two bone nodes in the spatial domain, and a temporary edge is connected to each other in a continuous time step. On this basis, the author constructs the graph convolution of multilayer space and time to combine the length information of the graph with the time information, which greatly improves the recognition rate of the network [24]. Some scholars proposed an end-to-end framework called the memory network as the center to enhance the spatial and temporal features of foot bone feature recognition. In the framework of the model, the module is temporarily modified to redefine the time focus of the bone wheel of the action line, and the powerful space-time convolution module of CNN is used to redefine the space-time relationship of human activities. It can obviously improve the accuracy of skeleton-based action recognition. Based on the above discussions, we give the main contributions of this work.

1. In this paper, the deep learning model is applied to the extraction and analysis of foot bone features for the first time, and good experimental results have been achieved
2. In this paper, the multiobjective optimization algorithm is used to select the optimal model parameters and further improve the performance of the model, so it has good theoretical value and application prospect

The article "Extraction and Analysis of Foot Bone Shape Features Based on Deep Learning" was published in 2022. Journal: Comput Math Methods Med.

## 3. Optimized CNN for Extraction and Analysis of Foot Bone Shape Features

### 3.1. Deep CNN Model Introduction

CNN adds the convolution layer and pooling layer to form the deep CNN model, which is shown in Figure 1.

The calculation process of convolution is shown below:

(1) $$\begin{array}{c} {\text{CONV}}_{\left(ij\right)}=\overset{m-1}{\underset{i}{\sum }}\overset{n-1}{\underset{j}{\sum }}u_{ij}\times w+b\;\left(i=1,2\cdots m-1,\;j=1,2\cdots n-1\right), \end{array}$$

where *u*_*ij*_ is the input image, *m* and *n* are the size of the input image, *w* is the size of the convolution kernel, and *b* is the bias constant of the convolution kernel. CONV (*ij*) is the characteristic graph output after convolution operation.

CNN adds an activation function layer to the network and analyzes the model better by adopting the feature mapping method of nonlinear function. Then, the mathematical expression of common activation function is introduced one by one as

(2) $$\begin{array}{c} f\left(x\right)=\frac{1}{1+e^{-x}}. \end{array}$$

In addition to the above activation functions, other common activation functions are as follows: the mathematical expression of tanh function is

(3) $$\begin{array}{c} f\left(x\right)=\frac{e^{x}-e^{-x}}{e^{x}+e^{-x}}. \end{array}$$

The mathematical expression of ReLU function is

(4) $$\begin{array}{c} f\left(x\right)=\max\left(0,x\right). \end{array}$$

The full name of the ReLU function is the rectified linear unit. The function is one of the commonly used activation functions, which is characterized by low computational complexity and no exponential operation. However, it is worth explaining that ReLU function has certain defects in the calculation process. When the data passes through the negative range of ReLU function, the output value is equal to 0. The Leaky-ReLU function can solve the above problem:

(5) $$\begin{array}{c} f\left(x\right)=\left\{\begin{array}{cc} x, & x\geq 0,\\ \alpha x, & x<0. \end{array}\right. \end{array}$$

The corresponding equations of sig and tanh are as follows:

(6) $$\begin{array}{c} \left\{\begin{array}{c} \text{sig}\left(x\right)=\frac{1}{1+\exp\left(-x\right)},\\ \tanh\left(x\right)=\frac{\exp\left(x\right)-\exp\left(-x\right)}{\exp\left(x\right)+\exp\left(-x\right)}, \end{array}\right.\\ h_{w,b}\left(x_{i}\right)=\left[\begin{array}{c} p\left(y_{i}=1\left|x_{i};w,b\right.\right)\\ p\left(y_{i}=2\left|x_{i};w,b\right.\right)\\ p\left(y_{i}=3\left|x_{i};w,b\right.\right)\\ \cdots \\ p\left(y_{i}=n\left|x_{i};w,b\right.\right) \end{array}\right]=\frac{1}{\sum_{j=1}^{n}e^{w_{j}x_{i}+b_{j}}}\left[\begin{array}{c} e^{w_{1}x_{i}+b_{1}}\\ e^{w_{2}x_{i}+b_{2}}\\ e^{w_{3}x_{i}+b_{3}}\\ \cdots \\ e^{w_{n}x_{i}+b_{n}} \end{array}\right]. \end{array}$$

The cross-entropy (CE) formula is as follows:

(7) $$\begin{array}{c} \text{loss}=-\frac{1}{m}\overset{m}{\underset{j=1}{\sum }}\overset{n}{\underset{i=1}{\sum }}y_{ji}\log\left({\hat{y}}_{ji}\right). \end{array}$$

The original form of the gradient descent method is shown below:

(8) $$\begin{array}{c} \theta ≔\theta -\alpha \frac{\partial }{\partial \theta }J\left(\theta \right). \end{array}$$

The mathematical expression of a common Adam optimizer is given as

(9) $$\begin{array}{c} m_{t}=\beta_{1}m_{t-1}+\left(1-\beta_{1}\right)g_{t},\\ v_{t}=\beta_{2}v_{t-1}+\left(1-\beta_{2}\right)g_{\text{t}}^{2}. \end{array}$$

The article "Extraction and Analysis of Foot Bone Shape Features Based on Deep Learning" was published in 2022. Journal: Comput Math Methods Med.

### 3.2. Optimized CNN Model

Since conventional CNNs are prone to local optimality, particle swarm optimization (PSO) is simple and easy to solve, but it is prone to local extreme points, low accuracy, slow convergence, and stagnation. In this section, the differential perturbation is introduced into the PSO to form the differential perturbation particle swarm optimization (DPPSO) algorithm, which makes use of the advantages of fast convergence speed and good global performance of difference, overcomes the shortcomings of low precision and local optimality caused by the use of PSO, and builds an optimized CNN model. The multiobjective optimization model is

(10) $$\begin{array}{c} \begin{array}{c} \min f_{1}\left(x_{1},x_{2}\right),\\ \max f_{2}\left(x_{1},x_{2}\right)\\ \begin{array}{c} \text{s}.\text{t}.\;p_{1}<g_{1}\left(x_{1},x_{2}\right)<q_{1}\\ p_{2}<g_{2}\left(x_{1},x_{2}\right)<q_{2}\\ p_{3}<g_{3}\left(x_{1},x_{2}\right)<q_{3}\\ p_{4}<g_{4}\left(x_{1},x_{2}\right)<q_{4}, \end{array} \end{array}\\ 120<x_{1}<180,\\ 120<x_{2}<180, \end{array}$$

where *f*_1_ represents energy consumption target, *f*_2_ represents the output target, and *g*_1_, *g*_2_, *g*_3_, *g*_4_ represent the packaging quality of 4 indicators: crushing strength, wear strength, drop strength, and compressive strength, respectively. It is worth noting the fusion mechanism of deep learning and differential perturbation particle swarm optimization (DPPSO) algorithm can be seen in Figure 2.

Based on the above discussions, the optimized deep neural network and its application in extraction and analysis of foot bone shape features are shown in Figure 2. It mainly includes data preprocessing, CNN model training and testing, and DPPSO algorithm design, finally getting the optimal model performance.

The article "Extraction and Analysis of Foot Bone Shape Features Based on Deep Learning" was published in 2022. Journal: Comput Math Methods Med.

## 4. Experimental Results and Analysis

### 4.1. Experimental Data Introduction

In recent years, human bone recognition technology has developed rapidly. Many researchers at home and abroad have carried out the research and application of human behavior recognition in different scenarios. Although there are differences in database and behavior recognition model, human behavior recognition technology is similar. The database in this paper mainly comes from depth sensors. The pixel value in the depth data represents the depth value, which is used to represent the distance between the camera and the object. The larger the value, the darker the distance will appear in the image. The smaller the value, the smaller the distance, and the brighter the display.

Firstly, the motion sequence is obtained by a sensor and then preprocessed by a computer (such as gray-scale morphological processing and denoising). Then, some coding mode is used to write the preprocessed data to describe its action characteristics. Finally, a classifier is used to train and test behavior categories, among which data acquisition and data pretreatment belong to the category of data pretreatment, and feature extraction behavior classification and understanding belong to the category of pattern recognition. In this paper, bone data from MSR-Action3D, UTkinect-Action, and Flerence3D-Action databases were used in the experiment. It is worth noting that the framework system of the CNN model applied in this paper is shown in Figure 3.

### 4.2. Experimental Result Analysis

In order to obtain more comprehensive information on foot bone, according to the human anatomy and the distribution of foot pressure, the human sole was divided into regions, and flexible pressure measuring units were placed in these regions to form a multisensor foot pressure detection system. Within a gait cycle, the statistical variation of pressure signals in different areas is shown in Figure 4.

In a complete gait detection cycle, the pressure sensor of the multipoint array can only collect the foot pressure signals of local corresponding regions in different gait periods due to the influence of the special touch form of the foot. For example, the sensor in the heel area can only record the pressure signal during the gait touching the ground, but when the heel leaves the ground, it cannot continue to collect the pressure signal effectively. A similar situation exists in other sensors. At the same time, the overlap between the signal and redundancy also increases the detection system in the burden of data transmission, processing, and storage; for the foot, eight areas of the pressure sensor have optimized configuration and are made with the best sensor array location with the least number of sensors, to maximize the amount of information limited to collect signals and finally get the ideal detection results.

The article "Extraction and Analysis of Foot Bone Shape Features Based on Deep Learning" was published in 2022. Journal: Comput Math Methods Med.

This paper also compares the graph convolutional network (GCN) before and after optimization, and the experimental database and sample selection are consistent with the previous section. The optimized GCN network contains 10 layers, including 64 convolutional kernels in layers 1 to 4, 128 convolutional kernels in layers 5 to 7, and 256 convolutional kernels in the last three layers. The stride of the five and eight layers is 2, and the default value of the other layers is 1. Finally, a whole office mean pooling was connected to softmax for classification, and the learning rate was set to 0.001, and the equal interval descent method was adopted to adjust the learning rate gamma value to 0.1. The dropout value was set to 0.5, the random loss information source was prevented from overfitting, and the batch size was set to 16. Cross-entropy was still selected as the loss function evaluation, and the random gradient descent (SGD) method was used for learning optimization.  Figure 5 shows the trend of feature extraction accuracy of the CNN model before and after optimization with the number of cycles. It can be seen from Figures 5(a) and 5(b) that the network reaches saturation accuracy at about 60 cycles, and the final accuracy is higher than that of the improved CNN.

Figure 6 shows the confusion matrix diagram of feature classification of the optimized CNN model in the data sets MSR-Action3D and UTkinect-Action. As can be seen from the figure, the feature classification accuracy of the model is different for different action subsets. However, no matter in which data set, the method proposed in this paper can achieve higher accuracy of feature classification. Thus, the stability and effectiveness of the proposed method for foot bone feature extraction are verified.

In order to further demonstrate the feature extraction accuracy of the proposed method, Figure 7 shows the relationship between classification accuracy and iteration times of different methods. We can figure out from the figure, with the increase in the iteration number, that the classification performance of the three methods shows an increasing trend. When the iteration number is 1200, the three models all reach the highest classification accuracy, which is 81%, 86%, and 98%, respectively. Therefore, the improved CNN model in this paper achieves the highest feature extraction accuracy. In addition, even when the number of iterations is small, the proposed method also has the best model performance throughout the training process, which demonstrates the effectiveness of the proposed method in the foot bone feature extraction field.

The article "Extraction and Analysis of Foot Bone Shape Features Based on Deep Learning" was published in 2022. Journal: Comput Math Methods Med.

In order to further show the characteristics of various features, Figure 8 shows the change of recognition accuracy of the proposed method in 18 action categories with respect to three features. The abscissa is 18 action categories, and the ordinate is the recognition accuracy. It can be found from the bar chart that different features in different action categories have good and bad recognition results. From the above observation, it can be found that motions with small amplitude and local concentration can be better discriminated by feature positions, motion tracks the bone node and motion lasting for a long time, and motions with feature motions can provide better representation. Feature bones have a relatively good recognition effect when it comes to local joint changes. The above experimental structures indicate that different bone structures may be represented by different features, and diversified features will provide richer information for bone structure discrimination. It also indicates the complementarity between different characteristics. Therefore, the above experimental results verify that it is reasonable to extract multiple features to comprehensively characterize a skeletal action in this paper.

To be noted, the classification results obtained by different methods are shown in Figures 9(a)–9(d). Specifically, there are plenty of overlaps between feature 1 (f1), feature 2 (f2), and feature 5 (f5) in Figure 9(a), which means the SVM cannot separate the three features well. And the similar situation happens in Figures 9(b) and 9(c). In contrast, from the visual results in Figure 9(d), we know that the optimized CNN method shows no overlaps in separating the three features, which means the optimized CNN achieves the best classification performance with the least misclassification points.

## 5. Conclusions

Nowadays, artificial intelligence and computer vision technology are widely developed, and bone feature extraction, as an important branch of computer vision, is widely used in intelligent video surveillance, robot vision, and other fields. Previous work is either based on static image of human skeleton recognition, or based on the continuous motion recognition of traditional video, each frame of image background segmentation manual extraction of human backbone, and then to identify and learn, the process is too complicated, and large amount of calculation.

The article "Extraction and Analysis of Foot Bone Shape Features Based on Deep Learning" was published in 2022. Journal: Comput Math Methods Med.

In view of the above problems, this paper conducted in-depth research on the extraction and analysis of human foot bone features and proposed the foot bone feature and extraction model based on the improved CNN model. This method not only has good extraction ability of foot bone features but also achieves high fault classification accuracy. The feasibility of the proposed method in human motion monitoring is verified by experiments. Future research may need to add factors such as the individual body structure and dietary habits of research subjects, so as to further improve the accuracy of foot bone feature extraction and recognition.

## Figures and Tables

**Figure 1:** The typical schematic diagram of CNN neural network.

**Figure 2:** The framework of the CNN-based foot bone shape feature extraction and analysis method.

**Figure 3:** The CNN model setting in this paper.

**Figure 4:** Multisensor foot bone pressure acquisition signal.

**Figure 5:** Comparison of feature extraction accuracy of CNN before and after optimization.

**Figure 6:** The confusion matrix diagram of feature classification of the optimized CNN model in different data sets: (a) MSR-Action3D; (b) UTkinect-Action.

**Figure 7:** The relationship between the feature extraction accuracy and iteration times of different methods.

**Figure 8:** Multifeature histogram comparison.

**Figure 9:** Feature classification accuracy by (a) SVM, (b) BP, (c) CNN, and (d) optimized CNN.

## Data Availability

The experimental data used to support the findings of this study are available from the corresponding author upon request.
